The article "5G Edge Computing Enabled Directional Data Collection for Medical Community Electronic Health Records" was published in 2021. Journal: J Healthc Eng.

# 5G Edge Computing Enabled Directional Data Collection for Medical Community Electronic Health Records

**DOI:** 10.1155/2021/5598077

**Published:** 2021-07-22

**Authors:** Xiaoqiang Yan, Xiaogang Ren

**Affiliations:** ^1^The Affiliated Changshu Hospital of Soochow University (Changshu No. 1 People's Hospital), Jiangsu, 215500 Changshu, Suzhou, China; ^2^China University of Mining Technology, Jiangsu, 221116 Xuzhou, China

## Abstract

It is important to promote the development and application of hospital information system, community health service system, etc. However, it is difficult to realize the intercommunication between various information systems because it is not enough to realize the in-depth management of health information. To address these issues, we design the 5G edge computing-assisted architecture for medical community. Then, we formulate the directional data collection (DDC) problem to gather the EMR/HER data from the medical community to minimize the service error under the deadline constraint of data collection deadline. Moreover, we design the data direction prediction algorithm (DDPA) to predict the data collection direction and propose the data collection planning algorithm (DCPA) to minimize the data collecting time cost. Through the numerical simulation experiments, we demonstrate that our proposed algorithms can decrease the total time cost by 62.48% and improve the data quality by 36.47% through the designed system, respectively.

## 1. Introduction

Recently, the core role of smart medicine is the construction of hospital information platform based on electronic medical records and regional health information platform with resident's electronic health records [1]. Electronic health records [2] can improve the phenomenon of information asymmetry between doctors and patients and satisfy the demand-oriented development of medical service reform. The construction of electronic health records is the focus of future smart medicine [3], which can not only satisfy the diversity requirements of medical and health reform but also accelerate and strengthen the development of information technology in medical and health institutions. Recently, the vigorous development of information technology in China's medical and health industry has given birth to the vigorous development and application of hospital information system (HIS), community health service system (CHSS), and other information systems. However, it is difficult to realize the intercommunication between various information systems because it is not enough to realize the in-depth management of health information.

The National Health Commission of the People's Republic of China [4] is committed to promoting the 5G-assisted medical action project. On the basis of medical and health information, it can promote not only the implementation of hierarchical diagnosis and treatment but also the reform of public medical institutions and public health management mode. Then, 5G-assisted medical care aims to improve the efficiency of medical institutions and integrate high-quality medical resources such as electronic health records (EHRs) [5], overcoming the shortcoming of traditional medical services and enabling patients and improving the upgrading of traditional medical service mode.

The scientific and technological application of medical community [6] electronic health records have been attracting the attention of many researchers and enterprises. Reference [7] compared achievement of and improvement in quality standards for diabetes at practices using EHRs with those at practices using paper records. Reference [7] examined the effects of electronic health records on the safety of patients in medical facilities. Reference [8] analyzed the costs and benefits of EHRs in six community health centers (CHCs) that serve disadvantaged patients.

However, the above researches do not deeply study the requirements and data characteristics of medical community platform for EHR management. In terms of credibility, reliability, and real-time, it is necessary to deeply study the directional collection mechanism of archival data, such as large-scale mobile terminal sensing under 5G, diversified archival data collection, and archival information sharing under the medical community.

So, there are some major challenges as follows:

- The diversity and complexity of medical community seriously restrict the classification efficiency and marking accuracy of medical community electronic health records data, which affects the intelligent management efficiency of EHRs.
- The differences of medical level and service objects between different medical institutions in the medical community make the sharing of electronic records, which is an important basis for specialist collaboration, more complex. The low efficient and precision data sharing will seriously restrict the medical community's ability to solve major diseases, and it is difficult to form a complementary development mode.
- How to accurately and timely collect the data of medical community electronic health record management has become a difficult problem because it is difficult to predict which medical structure will produce what type of electronic health record data at what time.

Our key contributions can be summarized as follows:

- We design the 5G edge computing-assisted architecture for medical community.
- We formulate the directional data collection (DDC) problem to gather the EMR/HER data from the medical community with minimizing the service error under the deadline constraint of data collection.
- We design the data direction prediction algorithm (DDPA) to predict the data collection direction and propose the data collection planning algorithm (DCPA) to minimize the data collecting time cost.
- We conduct extensive simulations for the designed system and proposed algorithms. The results show that our proposed algorithms can decrease the total time cost by 62.48% and improve the data quality by 69.95% through the designed system, respectively.

The rest of the paper is organized as follows. We review the state-of-the-art research in Section 2. We design the 5G-assisted edge computing system in Section 3. We present the system model and formulate the DDC problem in Section 4. We design the intelligent data collection scheme with the assistance of random forest for solving the DDC problem in Section 5. We conduct the simulations in Section 6. We conclude this work in Section 7.

## 2. Related Work

The current situation of medical archives management in the medical community is discussed as follows. Reference [9] found the significant deficiencies in the practice of warfarin management and suggestive evidence that anticoagulation services can partially ameliorate these deficiencies. Reference [10] described a randomized trial of a program to identify and treat depression among high utilizers of general medical care. Reference [11] designed an intelligent archive management system by integrating 5G network and Internet of Things for smart hospitals. Reference [12] used the exome sequencing for infants in intensive care units to determine the diagnostic yield and use of clinical exome sequencing in critically ill infants. Reference [13] proposed a novel drug supply chain management using hyper ledger fabric based on block-chain technology to handle secure drug supply chain records.

About the status of data collection, reference [14] extracted security data that plays an important role in detecting security anomaly toward security measurement. Reference [15] provided a theoretical model of privacy in which data collection requires the consent of consumers who are fully aware of the consequences of consent. Reference [16] considered a scenario where an unmanned aerial vehicle collects data from a set of sensors on a straight line. Reference [17] proposed a low redundancy data collection scheme to reduce the delay as well as energy consumption for monitoring network by using matrix completion technique. Reference [18] proposed a practical framework called *Privacy Protector*, patient privacy-protected data collection, with the objective of preventing these types of attacks.

## 3. 5G-Assisted Edge Computing System

First of all, according to the requirements of medical community e-health records management, based on the complex environment of regional medical institutions information platform, we design the mathematical model of e-health records management and its 5G application system framework. Secondly, by deploying multiple mobile terminal nodes, we design the medical community electronic health records management 5G architecture, to provide real-time and reliable communication guarantee for large-scale medical community electronic health records data application business. Then, in order to ensure the real-time and reliability of data sharing of medical community electronic health records, a massive data collection mechanism based on edge computing is established. Finally, based on the above requirements, we combine the large-scale mobile communication of 5G with the massive data real-time collection technology of edge computing to study the application mechanism of data directional collection, so as to provide the reliability, credibility, and feasibility guarantee for the data update and sharing application of medical community electronic health records management.

According to the requirements of regional medical institutions information platform construction, we analyze the information interconnection and regional differences between community health service centers and municipal hospitals. Then, we introduce edge computing into 5G through the organic allocation and deep integration between the mobile terminals and cloud computing server. The edge computing reasonably allocates the storage, computing, and network services resources between the computing center and the mobile terminals, so as to achieve the local optimal division of labor and cooperation before the network service quality and user experience quality. Therefore, the introduction of edge computing into 5G can satisfy the computing and communication needs of mobile terminals with distributed and random characteristics. Hence, edge computing can well solve the geographical deployment characteristics of 5G nodes scattered between community health service centers and municipal hospitals. Moreover, the edge computing architecture with 5G is shown in Figure 1. Here, the 5G platform is the center, i.e., the municipal hospital, and several subnets of edge community service center are deployed. The network control ability of these center subnets is the same as that of the servers in the platform, where the architecture can effectively reduce the calculation delay and improve the storage efficiency of medical community electronic health record data.

The 5G architecture shown in Figure 1 can provide convenient services, health management services, traditional Chinese medicine (TCM) health care services, and other services. This architecture can give full play to its advantages in data sharing and family doctor follow-up, continuously improve the accessibility and effectiveness of services, comprehensively improve service level and satisfaction, and provide medical services and health management services to the majority of residents conveniently and quickly. At the same time, the medical community platform can solve the following problem, lack of medical resources shortage, difficulty to see a doctor, and realize the integration of health resources and then improve the level of primary health care through the establishment of complete electronic health records for residents. Then, we integrate the sharing of medical records and test results, medical images, medication records, and patients' basic health information between secondary and tertiary comprehensive medical institutions in the community to realize the sharing of high-quality medical resources in the region.

With the rapid development of 5G edge terminals used to collect electronic health records data, how to reasonably allocate and effectively recover the diversity resources of 5G has become a key problem. In 5G environment, the distribution and recovery of resources and the reconstruction of network topology are dynamic. There is an unknown mapping and interference relationship between 5G real-time resource statistics, computing task resource allocation and task scheduling, and 5G network edge computing terminal trusted resource information. These relationships are real-time and random. It is the main goal of network resource management to make 5G system execution efficiency and resource utilization always in the best state. It is well known that 5G supports a large amount of traffic. The resource request queue is very easy to overflow, which makes the arrival rate and processing efficiency of resource request signaling and computing task control signaling between the network control center and the edge terminal irregular, and the reliability of resource allocation and computing task unbalanced among different services. In order to improve the instantaneous resource management level of 5G and the utilization rate of global resources and make 5G better communication support for medical community electronic health records management, we design the 5G edge computing architecture as shown in Figure 2, where we deployed with multiple edge terminals, multiple autonomous base stations, and multiple autonomous control networks.

In Figure 2, edge computing terminals share EHR information and exchange unified standard data sources through regional platform interfaces of medical institutions. According to the edge computing architecture shown in Figure 2, medical institutions improve the interconnection architecture of regional health information platform and guide the electronic medical record system and electronic health record management system of medical institutions under their jurisdiction. In particular, electronic health records need to achieve unified data interface standards of medical institutions, medical insurance, community, and other related systems, so as to facilitate information sharing.

The common data element established in the 5G control center of medical community can efficiently improve the real-time sharing efficiency of electronic medical record (EMR) and EHR. Therefore, the electronic medical records and electronic health records storage system of medical institutions in medical community must follow the standardized description of national public health data element attributes, describe the extracted data element attributes, conduct business modeling, and realize data sharing. Medical institutions at all levels should use the ID number as the main identification code for the transmission and circulation of information in the diagnosis and treatment of public health services in the business system, so as to ensure the effective collection of archival information. Each edge computing terminal server should ensure the validity and timeliness of data transmission, verification, process tracking, and traceability, so as to ensure that all kinds of information can be uploaded to 5G information platform timely, accurately, and comprehensively.

Therefore, how to collect and improve data from the community and medical institutions at all levels in accordance with the electronic medical record information standards and unified specification of disease coding and other important databases, to ensure the quality of data, has become the key of medical community archives management. The process of data collection should have the following properties:

- The process of data collection should be based on the main index of patient identity, correctly associated with the previous diagnosis and treatment data, and form a complete and standardized medical record file, which is convenient for medical staff to use.
- The process of data collection should be carried out according to the interface specification of regional information platform. The diagnosis and treatment information should be uploaded and collected into health records in time.
- The process of data collection should implement the codes of clinical symptoms, diagnosis, surgery, drugs, inspection, and so on released by the state to ensure the standardization and unification of diagnosis and treatment information uploaded to the platform.

Figure 3 gives a toy example for the Directional Data Collection and application of medical community electronic health record with the above characteristics. In this scenario, cloud platform, edge computing terminal, and 5G platform are effectively integrated into the directional data collection of medical community electronic health records, such as community classification, data directional collection, and data storage.

The edge computing procedure is illustrated as follows:

1. The communities generate their EMR/HER data, which can be collected by a corresponding opportunistically encountered edge computing terminal.
2. The edge computing terminal analyzes and mines the valid information from collected EMR/HER data, e.g., the location, resident ID, and his/her historical records. Then, the dataset is sent to the cloud servers in real time. The edge computing terminal predicts their medical demand according to the historical records by using the algorithm proposed in Section 4.1 and returns the prediction results to the 5G cloud servers.
3. The 5G cloud servers periodically compute the data collection route via the algorithms in Section 4.2 for data collection terminal according to the information of communities and residents from edge computing terminals.
4. The data is collected by the data collection terminal through the route calculated in the above step.

## 4. Directional Data Collection for Medical Community

### 4.1. System Model

Suppose that the 5G platform of medical community includes *m* medical institutions and *n* communities. According to the scope of service and medical level, the mapping relationship between each community and different medical institutions is established, denoted by *C*={*c*_*ij*_}_*i*=1,*j*=1_^*m*,*n*^. Here, the electronic file data is generated by the medical institutions according to the community it serves, which is used to obtain the medical needs and feedback of residents. Note that each medical institution initiates one data collection task in the time dimension. So, *T*={*t*_*i*_}_*i*=1_^*m*^ denotes the task set. For convenience, we define the data collection process as follows.

**Definition 1 (data collection task).**

The process of edge computing terminal completing data collection task is to select the corresponding observation values from a series of candidate data samples corresponding to the community for 5G platform.

For each data collection task *t*_*i*_, we assume that it has a candidate sample set *A*_*i*_ shown as follows:

(1) $$\begin{array}{c} A_{i}=\left\{a_{i}\left(1\right),a_{i}\left(2\right),\ldots ,a_{i}\left(\left|A_{i}\right|\right)\right\}. \end{array}$$

Then, let *a*_*i*_(0) denote the optimal data sample corresponding to the task *t*_*i*_. Therefore, the data error caused by task *t*_*i*_ can be calculated by

(2) $$\begin{array}{c} e_{i}=\frac{1}{\left|A_{i}\right|}\left(\sum_{k=1}^{\left|A_{i}\right|}a_{i}\left(k\right)-a_{i}\left(0\right)\right). \end{array}$$

The resident set who provides the EMR/HER dataset from all communities can be represented as follows:

(3) $$\begin{array}{c} B_{i}={\left\{b_{i}^{j}\right\}}_{j=1}^{n}. \end{array}$$

Here, *b*_*i*_^*j*^ represents the data in task *t*_*i*_, which is provided by the *j*-th community when the *i*-th task is initiated by *i*-th medical institution when there is the mapping relationship belonging to *C*. So, we can calculate the data matrix corresponding to data collection tasks from all communities through the following equation:

(4) $$\begin{array}{c} A={\left\{a_{ij}\right\}}_{i=1,j=1}^{m,n}\\ =\prod_{i=1}^{m}\left(A_{i}-e_{i}B_{i}\right)\\ =\prod_{i=1}^{m}\left(\overset{\left|A_{i}\right|}{\underset{k=1}{\sum }}\int a_{i}{\left(k\right)}^{t}\text{d}t-e_{i}B_{i}\right)\\ =\prod_{i=1}^{m}\left(\overset{\left|A_{i}\right|}{\underset{k=1}{\sum }}\int a_{i}{\left(k\right)}^{t}\text{d}t-e_{i}\overset{n}{\underset{j=1}{\sum }}b_{i}^{j}\right). \end{array}$$

Here, we redefine the data sample *a*_*i*_(*k*) in *A*_*i*_ as *a*_*i*_(*k*)^*t*^, which is calculated according to the time dependence of edge computing. Note that we can update the mapping relationship between each community and different medical institutions through the following equation:

(5) $$\begin{array}{c} c_{ij}=\left\{\begin{array}{cc} 0, & \text{if }0<\frac{a_{ij}}{e_{i}}<\gamma_{ij},\\ 1, & \text{if }\frac{a_{ij}}{e_{i}}\geq \gamma_{ij}. \end{array}\right. \end{array}$$

Here, *γ*_*ij*_ is the tolerance threshold of the data collection error, which is a given empirical value.

In order to analyze the direction accuracy of data collection conveniently, we give the following definition of data collection aggregation reliability.

**Definition 2 (data collection task).**

For *m* data collection tasks and *n* communities, the direction of data collection is accurate when each task satisfies the following conditions:

(1) The *i*-th task and *j*-th community have the mapping relationship, i.e., *c*_*ij*_=1.
(2) *A*_*i*_ and *B*_*i*_ have the same rank for each task *t*_*i*_.
(3) All the data samples collected by all the medical institutions have consistency; i.e., the following function *f*(*A*) is valid:
  (6) $$\begin{array}{c} f\left(A\right)=\underset{n⟶\infty }{\lim}\frac{\lim_{m⟶\infty }A}{\sum_{i\prime =1}^{i}r_{i}^{\prime }+\sum_{e\in T_{i}}t_{e}}. \end{array}$$
(4) Let Γ(*t*_*i*_) denote the data collection time cost. The time cost of the *i*-th task is not larger than the deadline *τ*_*i*_.

### 4.2. Problem Formulation

The objective of directional data collection (DDC) problem is to design a data collection scheme based on 5G edge computing system to gather the EMR/HER data from the medical community to minimize the service error under the deadline constraint of data collection. *x*_*ij*_ is a binary variable to indicate whether data of task *t*_*i*_ is collected from *j*-th community. *x*_*ij*_=1 if data of task *t*_*i*_ is collected from *j*-th community. *x*_*ij*_=0 otherwise.

The DDC problem can be formulated as follows:

(7) $$\begin{array}{c} \text{DDC }\min\;x_{ij}\overset{m}{\underset{i=1}{\sum }}e_{i}\\ \text{s.t.}\;\begin{array}{c} \left(\text{a}\right)\;x_{ij}\in \left\{0,1\right\},\;\forall t_{i}\in T;\\ \left(\text{b}\right)\;r\left(A_{i}\right)=r\left(B_{i}\right),\;\forall t_{i}\in T;\\ \left(\text{c}\right)\prod_{i=1}^{m}\prod_{j=1}^{n}c_{ij}=1;\\ \left(\text{d}\right)\;\Gamma \left(t_{i}\right)\leq \tau_{i},\;\forall t_{i}\in T. \end{array} \end{array}$$

Constraint (a) gives the value range of *x*_*i*,*j*_. Constraint (b) ensures that the rank of candidate data sample set is equal to that of data in task *t*_*i*_ on the basis of *C*. Constraint (c) ensures that each mapping between the task and its corresponding community is valid. Constraint (d) ensures that the time cost of data collection in each task is not larger than its deadline.

We list the frequently used notations in Table 1.

## 5. Intelligent Data Collection Scheme

In this section, we propose our 5G edge computing enabled directional data collection (5EDDC) algorithm. Then, the detailed description of the proposed algorithm is presented in two phases: data direction prediction and data collection planning.

### 5.1. Data Direction Prediction Algorithm

Medical behaviors and requirements of residents in different communities actually reflect the regeneration direction of EMR, which contains a lot of medical information, such as common diseases and medical habits. Based on the implementation of a variant of algorithms [19], we design Algorithm 1 for solving the problem of data direction prediction.

First, we predict the medical behavior of residents through the following steps:

 
*Step 1. Feature extraction* takes into account the following features for each behavior in community generating along the historical records *B*_*i*_ with the last data collection task *t*_*i*_ and candidate sample set *A*_*i*_ of current medical community: time of day, medical behavior starting time, medical community name and its location, resident ID, and medical treatment time of each location. The above procedure is denoted as function Feature Extraction(dataset).
 
*Step 2. Random forest-based prediction* needs the input vector *n*_*t*_ representing the information of a resident, which includes the origin community and destination medical institute, as well as the corresponding extracted features from step 1. Then, the data generating time of any community can be predicted based on temporal data dependencies and spatial data correlations. The above process is denoted as function Random Forests.

Second, we can predict the data direction of community for collecting data via the Interval-based Historical Average (IHA) [20] as shown in the following equation:

(8) $$\begin{array}{c} \text{IHA}\left(E\left[t_{a}\right],\lambda \right)=\frac{1}{2\lambda +1}\sum_{p=-\lambda }^{\lambda }\left(\sum_{q=1}^{\text{days}}\left(t_{p}-E\left[t_{a}\right]-q\right)\right). \end{array}$$

Here, *E*[*t*_*a*_] is the expectation of data generating time of task *t*_*a*_ based on historical EMR/HER data, *λ* is the mean absolute error of the random forests [21] for data generating time prediction, and days is the days of historical EMR/EHR dataset. *t*_*p*_ is the first data collection starting time after *E*[*t*_*a*_]+*q* in the *p*-th day of the dataset, where *E*[*t*_*a*_]+*q* is the generating time of EMR/HER data for recording residents in *a*-th community at the *q*-th day. Thus, *t*_*p*_ − *E*[*t*_*a*_] − *q* is the historical data collection time on the *q*-th day. Finally, we calculate the EMR/EHR data generating time of communities and data collection direction of medical community.

In Algorithm 1, the Sink(*F*, *B*) function is used to find all the data collection sinks of EMR/EHR at its medical community. In addition, Algorithm 1 updates all the data samples and records between any two communities and computes their collecting time through the following steps:

1. Find all ${\bar{a}}_{i}$, which can satisfy the tolerance
2. Extract all the features from historical dataset

### 5.2. Data Collection Planning Algorithm

Based on the direction prediction of data collection, the DDC problem is equivalent to finding a data route to collect the EMR/HER data for all selected medical communities with minimum time cost. The above data collection planning (DCP) problem can be formulated as follows:

(9) $$\begin{array}{c} \text{DCP }\min\sum_{0=1}^{C}\Gamma \left(t_{o}\right). \end{array}$$

Moreover, we design the data collection planning algorithm (DCPA) to solve the DCP problem. The basic idea is given as follows (see Algorithm 2):

1. Transform *A*_*i*_ and integrate into $\tilde{A}$ (line 5)
2. Update $\tilde{B}$ (line 6)
3. For each element in $\tilde{B}$, we first divide it into two separate sets *P*_1_ and *P*_2_, and then remove half of elements in $\tilde{B}$ (lines 8–10), and then find the corresponding subroutes (lines 11–14)
4. Integrate all the subroutes into the final data collection planning *P* (lines 15–18) where the symbol ⊎ represents the integration of some routes.

## 6. Numerical Experiments

In this section, we conduct extensive simulations to verify the performance of our proposed algorithms with different number of medical institutions, number of communities, days of month, and number of residents of a community.

### 6.1. Data Description

The dataset used in our experiments is from the electronic records system of Changshu No. 1 People's Hospital. The dataset shows a kind of representative medical community data. It is generated by the medical community supported by Changshu No. 1 People's Hospital, which covers the period from January 1, 2018, to November 30, 2018. The dataset includes the record data of medical institute and residents, and GPS data of medical institutes. The data record contains various fields, such as time of day, medical behavior starting time, medical community name and its location, resident ID, medical treatment time of each location, and the number of patients of the corresponding medical institute, etc. The GPS data contains latitude, longitude, and treatment time of medical institute.

### 6.2. Simulation Setup and Benchmark

We assume that there are 10 medical institutions to provide medical care for 10 communities, which are supported by Changshu No. 1 People's Hospital. The residents receive medical treatment from the above medical institutions. In our simulation, we evaluate the total time cost of data collection, and data quality calculated by equation (2). All the simulations were run on a cloud server ECS [23] with 12-core Intel Xeon Platinum 8269CY and 48 GB memory. The other parameter settings of our simulations are listed in Table 2.

We develop the data collection algorithm DCA in [22] as the benchmark algorithm for comparison, which can make an efficient tradeoff between the data collection efficiency and energy consumption through the combination of the energy of the emotional device wireless device.

### 6.3. Performance Evaluation

In this subsection, we evaluate the performance of our algorithms and DCA in the scenario shown in Figure 4. Tables 3 and 4 give the locations of medical institutions and communities in the area, respectively. The above information is calculated based on Google Maps.

Figure 5 shows the prediction errors on two different days, i.e., March 10, 2018, and October 20, 2018. The prediction results demonstrate the effectiveness of our proposed prediction algorithm DDPA. The average prediction error on March 10, 2018, and October 20, 2018, is 3.21% and 1.93%, respectively.

Figures 6 and 7 show the impact of medical institutions on total time cost and data quality of our algorithms and DCA, respectively. The average total time cost of our algorithms and DCA is 8.85 hours and 2.44 hours, respectively. The average data quality of our algorithms and DCA is 75.76% and 94.75%, respectively. The results show that our algorithms can reduce 72.38% of total time cost of DCA on average, and improve 25.06% of data quality of DCA, respectively. This indicates that the proposed algorithms significantly outperform DCA. This is because the data quality of our algorithms is better than the those obtained by DCA, respectively.

Figures 8 and 9 show the impact of communities on total time cost and data quality of our algorithms and DCA, respectively. The average total time cost of our algorithms and DCA is 5.75 hours and 1.63 hours, respectively. The average data quality of our algorithms and DCA is 73.27% and 97.59%, respectively. The results show that our algorithms reduces 71.67% of total time cost of DCA on average, and improves 33.20% of data quality of DCA, respectively.

Figures 10 and 11 show the impact of days of month on total time cost and data quality of our algorithms and DCA, respectively. The average total time cost of our algorithms and DCA is 16.15 hours and 9.99 hours, respectively. The average data quality of our algorithms and DCA is 63.31% and 94.01%, respectively. The results show that our algorithms can reduce 38.12% of total time cost of DCA on average, and improve 48.49% of data quality of DCA, respectively.

Figures 12 and 13 show the impact of communities on total time cost and data quality of our algorithms and DCA, respectively. The average total time cost of our algorithms and DCA is 8.92 hours and 2.86 hours, respectively. The average data quality of our algorithms and DCA is 68.44% and 95.21%, respectively. The results show that our algorithms can reduce 67.76% of total time cost of DCA on average and improve 39.11% of data quality of DCA, respectively.

Overall, our algorithms can significantly decrease the total time cost and improve the data quality through the designed data direction prediction algorithm and data collection planning algorithm.

## 7. Conclusion

In this article, we have designed the 5G edge computing architecture for medical community to improve the effectiveness and efficiency of EMR/EHR data collection. First, we formulate the directional data collection (DDC) problem to gather the EMR/HER data from the medical community for minimizing the service error under the deadline constraint of data collection deadline. Second, we design the data direction prediction algorithm (DDPA) to predict the data collection direction, and propose the data collection planning algorithm (DCPA) to minimize the data collecting time cost. Finally, through the numerical simulation experiments, we demonstrate that our proposed algorithms can decrease the total time cost by 62.48% and improve the data quality by 36.47% through the designed system, respectively.

## Figures and Tables

**Figure 1:** 5G architecture for medical community.

**Figure 2:** 5G edge computing architecture for medical community.

**Figure 3:** Application of directional data collection with the assistance of 5G and edge computing system.

**Figure 4:** Medical community for EMR/HER data collection. The red nodes represent locations of medical institutions and the green nodes represent locations of communities.

**Figure 5:** Prediction errors on March 10, 2018, and October 20, 2018.

**Figure 6:** Total time cost vs. number of medical institutions.

**Figure 7:** Data quality vs. number of medical institutions.

**Figure 8:** Total time cost vs. number of communities.

**Figure 9:** Data quality vs. number of communities.

**Figure 10:** Total time cost vs. days of month.

**Figure 11:** Data quality vs. days of month.

**Figure 12:** Total time cost vs. number of residents of a community.

**Figure 13:** Data quality vs. number of residents of a community.

**Algorithm 1:** Data direction prediction algorithm (DDPA).

**Algorithm 2:** Data Collection Planning Algorithm (DCPA).

**Table 1:** Frequently used notations.

Notation	Description
*c*_*ij*_	Mapping relationship between *i*-th community and *j*-th different medical institution
*C*	Set of mappings
*t*_*i*_	*i*-th data collection task
*T*	Set of tasks
*A*_*i*_	Set of candidate data samples belonging to *i*-th task
*a*_*i*_(*k*)	*k*-th data sample in *A*_*i*_
|*A*_*i*_|	Size of data sample in *A*_*i*_
*a*_*i*_(0)	Optimal data sample corresponding to task *t*_*i*_
*e*_*i*_	Data error caused by task *t*_*i*_
*b*_*i*_^*j*^	Data in task *t*_*i*_ provided by the *j*-th community when the *i*-th task is initiated by *i*-th medical institution
*B*_*i*_	Set of data in task *t*_*i*_ on the basis of *C*
*a*_*i*_(*k*)^*t*^	*k*-th data sample calculated according to the time dependence of edge computing
*γ*_*ij*_	Tolerance threshold of the data collection error between the *i*-th task and *j*-th community
*f*(*A*)	Consistence function
*τ*_*i*_	Deadline of task *t*_*i*_

**Table 2:** Parameter settings.

Parameter	Value
*n*	10
*m*	10
|*T*|	10
*γ*_*ij*_	[0.01, 0.05]
*τ*_*i*_	[1, 10] hours
|*A*_*i*_|	[100, 500]

**Table 3:** Locations of medical institutions.

*i*	Longitude	Latitude
1	31.629934025445163	120.74572694707317
2	31.637070592885376	120.74498723499269
3	31.641308857555806	120.74260543350061
4	31.644304755694158	120.743120417607
5	31.639559503878488	120.73996684991539
6	31.63350810894618	120.74108193885252
7	31.634421579375328	120.73520253697116
8	31.640051243952147	120.74334217244697
9	31.63600474671818	120.74427558114591
10	31.640862982947134	120.74781351639375

**Table 4:** Locations of communities.

*i*	Longitude	Latitude
1	31.633639306384033	120.73640714235745
2	31.635638094098336	120.74413897983557
3	31.64162333734517	120.74648660051481
4	31.638983794798012	120.74880870356253
5	31.641820359193588	120.73842118763615
6	31.63745217402931	120.74375621572658
7	31.643893501251643	120.74744351115115
8	31.63659402090503	120.742072053155
9	31.634475760812066	120.74353931598635
10	31.634834238968633	120.74956147326746

## Data Availability

The labeled dataset used to support the findings of this study is available from the corresponding author upon request.
